# Effects of Sacubitril/Valsartan on the Expression of CaMKII/Ca_v_1.2 in Atrial Fibrillation Stimulation Rabbit Model

**DOI:** 10.1155/2022/5832543

**Published:** 2022-07-28

**Authors:** Qi Lou, Lu-yi-fei Li, Guang-zhong Liu, Cheng-chuang Zhan, Li Zhang, Yan-xiang Zang, Wei-min Li

**Affiliations:** ^1^Department of Cardiology, First Affiliated Hospital of Harbin Medical University, Harbin 150001, China; ^2^Department of Cardiology, Shenzhen People's Hospital, Shenzhen 518020, China; ^3^Department of Cardiology, First Affiliated Hospital of Soochow University, Soochow 215006, China

## Abstract

**Methods:**

Overall, 18 rabbits were randomly divided into control, pacing (600 beats/min), and pacing+sac/val groups. The rabbits in the pacing+sac/val cohort received oral sac/val (10 mg/kg twice daily) across the 21-day investigation period. After three weeks, the atrial effective refractory period (AERP) and AF induction rate were compared. HL-1 cultures were exposed to fast pacing (24 h) with and without LBQ657 (active sacubitril form)/valsartan. Western blots were used for detecting Ca_v_1.2 and CaMKII expression within atrial muscles of the rabbits and HL-1 cultures of AF model.

**Results:**

In comparison to the sham cohort, the AF induction rate was markedly increased together with AERP reduction within pacing cohort. Such changes were markedly rescued through sac/val treatment in pacing+sac/val cohort. The proteomic expression profiles of CaMKII and Ca_v_1.2 showed that the CaMKII expression was markedly upregulated, while Ca_v_1.2 expression was downregulated in the pacing cohort. Importantly, these effects were absent in pacing+sac/val cohort.

**Conclusion:**

Results of this study show that sac/val treatment regulates the expression of CaMKII/Ca_v_1.2 and could alter this pathway in atrial rapid electrical stimulation models. Therefore, this investigation could contribute to a novel strategy in AF therapeutics in clinical settings.

## 1. Introduction

Atrial fibrillation (AF) is the most common long-lasting heart rhythm abnormality in people who have heart failure (HF) which is linked to high morbidity and death rates, thus being a major challenge for modern-day societies/economies [1, 2]. Heart failure often coexists with AF because they share some common pathophysiologic mechanisms and risk factors. Atrial electrical remodeling and structural remodeling, together with autonomic remodeling, are responsible for AF pathogenesis/prolonged establishment [3, 4]. Electrical remodeling is usually an early manifestation of atrial remodeling [5]. Electrical remodeling for the atrium is mainly related to changes in ion channels within atrial myocytes, particularly the calcium channels. L-Type calcium channels (LTCCs) represent the most important pathway for extracellular calcium influx when cardiomyocytes are excited [6]. LTCCs have four subtypes including Ca_v_1.1, Ca_v_1.2, Ca_v_1.3, and Ca_v_1.4 where Ca_v_1.2 is present in the myocardium [7]. Ca_v_1.2 is the upstream protein that regulates L-type calcium current (*I*CaL). Ca_v_1.2 protein expression reduction results in a decrease in *I*CaL, which shortens action-potential duration (APD), eventually promoting the occurrence of arrhythmias such as AF [8].

Electrical remodeling caused by abnormal calcium regulation in atrial myocytes has a pivotal role in AF pathogenesis/establishment. CaMKII works as a serine/threonine kinase that can phosphorylate Ca_v_1.2 and induce abnormal calcium regulation in myocardial cells, exacerbating AF pathogenesis [9]. Epidemiology-based investigations demonstrated that the prevalence of AF is increasing each year and causing reduced quality of life because of insufficient treatment options [10]. Therefore, strategies for effective regulation of CaMKII/Ca_v_1.2 signaling pathway are needed to prevent and correct the electrical remodeling in AF.

Some studies have confirmed that the natriuretic peptide (NP) family can improve electrical remodeling [11], but the specific mechanism is unclear. Experimental studies have shown that valsartan can improve atrial electrical remodeling in AF [12]. Sacubitril/valsartan (sac/val) is a combination of an angiotensin receptor–neprilysin inhibitor (ARNi) drugs, given orally for treating HF. This combination is composed of an enkephalinase (sacubitril) and angiotensin-receptor antagonist (valsartan) linked by hydrogen bonds at a molar ratio of 1 : 1. The drug has dual regulatory effects; i.e., it can inhibit the renin-angiotensin-aldosterone system (RAAS) via antagonism of angiotensin II receptor 1 (AT_1_R). On the other hand, it can simultaneously inhibit the degradation of NPs, such as A-type NPs (ANPs), B-type NPs (BNPs), and C-type NPs (CNPs) through enkephalinase leading to increased levels of cyclic guanosine monophosphate and reduced cardiac remodeling in patients with heart failure (HF) [13–17]. Clinical studies have shown that the sac/val treatment is more effective than enalapril for lowering all-cause-/sudden cardiac-mortality rates in aggravated HF clinical cases having lowered ejection-fraction/s [18–20]. The sac/val combination is gaining wider research interests these days for various cardiac-related pathway regulation. In a recent study, it was shown to decrease AF susceptibility by inhibiting angiotensin II-induced AF through p-Smad2/3, p-JNK, and p-p38 signaling pathways [21]. In this study, we aim to validate sac/val influence on CaMKII/Ca_v_1.2 expression in rabbit model and HL-1 AF cultures.

## 2. Methods

### 2.1. Animal Model of Fast Atrial Pacing

This research was performed according to the directives of the Care and Use of Laboratory Animals (US National Institutes of Health; no. 85-23). The study protocol was approved by the Ethics Committee of Harbin Medical University. Healthy-adult, male New Zealand white rabbits (approximately 3 kg, four months old) were procured from the Experimental Animal Center affiliated with the First Affiliated Hospital of Harbin Medical University. All the animals were housed in a specialized, nonpathogenic laboratory animal center, in individual cages, and received *ad libitum* filtered water and diet. Rabbit-based models for rapid pacing were developed following previous research protocol [22, 23]. A surface electrocardiogram (ECG) was performed on the individual animal, whereby those animals that demonstrated baseline/normal sinus rhythm at investigation commencement were consequently anesthetized using xylazine (5 mg/kg, Sigma-Aldrich™, USA) and ketamine (35 mg/kg, Sigma-Aldrich™, USA). A pacemaker (Harbin Polytechnic University, Harbin, China) was placed within a subcutaneous (SC) pocket on the animal's dorsal region. A pacemaker electrode was stitched onto the right atrium of the animal heart. Animals were confined for seven days postpacemaker implantation surgery for recovery, followed by randomization into three cohorts (*n* = 6/cohort) including (1) control cohort (the rabbits underwent a sham operation, i.e., sutured electrode only) with no pacing, (2) pacing cohort (the rabbits received an electrode and underwent fast atrial pacing, i.e., 600 bpm/21 days), and (3) the pacing+sac/val cohort (the rabbits underwent fast atrial pacing, i.e., 600 bpm/21 days while receiving sacubitril/valsartan (Novartis Pharma Schweiz AG™, Switzerland) oral treatment of 10 mg/kg, twice daily for 21 days) [15].

### 2.2. HL-1 Culture Model of High-Frequency Electrical Stimulation

HL-1 cultures stemming from the murine atrial tumor (AT-1) cells are considered immortalized cultures. Differentiated HL-1 culture lines show cardiac morphological, biochemical, and electrophysiological functions similar to atrial cardiomyocytes [24, 25]. HL-1 cells were cultured in DMEM/low glucose (JRH Biosciences™, USA) augmented with 9% fetal calf serum and 0.9% penicillin-streptomycin solution (Gibco-BRL, Rockville, MD, USA). Six-well plates were used to culture HL-1 cultures (≥1,000,000 myocytes), and YC-2 program-controlled stimulator (Chengdu™, China) was used for 24 hours [23] with a 1.5 V/cm pulse voltage, a 5-millisecond square wave width and duration, and a frequency of stimulation of 10 Hz. The necessary capture-effectiveness approximated 90% of all HL-1 cultures across a stimulatory timespan. HL-1 cultures were split into three cohorts: (1) control cohort (receiving no stimulatory/pharmacological treatments, with 24 h culturing time), (2) the pacing cohort (received high-frequency field-stimulation (24 h) as described previously), and (3) the pacing + sac/val cohort (treated with high-frequency field-stimulation (24 h) + LBQ657 and valsartan (both at 10 *μ*mol/L; MedChem Express™, USA)) [26, 27].

### 2.3. AERP/AF Induction Rate Determinations

The rabbits' atrial electrophysiological analyses were conducted according to previously published literature [22, 23]. Within such rabbits, the AERPs were registered using baseline cycle lengths (150 milliseconds), whereby eight essential stimuli (S1) and a subsequent premature stimulus (S2) were applied. The S1–S2 interval was extended (5 ms) and consequently lowered (2 ms-steps) until S2 failed in catching depolarization and consequently deemed as AERP (determined across three technical replicates for a mean AERP assertion). Consequently, AF induction involved the application of 10s pacing (10 Hz, 2 ms) onto the atrium using a fourfold present threshold current [28], with individual animals treated 10 times. The AF induction rate was determined by dividing AF times by induction times in each cohort [29].

### 2.4. Western Blot Assay

Proteomic specimens from the left atrial tissues were collected through animal atria/HL-1 cultures. Proteomic content was transferred to polyvinylidene fluoride membranes and analyzed through a proteomic assay kit (Bio-Rad™, Canada) via Western blotting following previously published literature [30]. The antibodies included CaMKII antibody (1 : 2000; Wanleibio, Shenyang, China), Ca_v_1.2 antibody (1 : 1000; Abcam™, China), and GAPDH antibody (1 : 10000; ZSGB-BIO™, China). Other antibodies were horseradish peroxidase-conjugated goat anti-rabbit (1 : 5000; ZSGB-BIO, China) and goat anti-mouse immunoglobulin G (1 : 3000; ZSGB-BIO™, China). The Western blot result bands were subjected to GAPDH-internal control normalization for comparison.

### 2.5. Statistical Analysis

SPSS® v.22.0 was used for all statistical analysis in this research. *P* < 0.05 was considered a statistically significant difference between results. All quantitative data were presented as mean ± standard error for mean, except for AF induction rate, which was presented as a percentage. The SNK-Q test based on one-way analysis of variance (ANOVA) was employed for the comparison of mean values.

## 3. Results

### 3.1. Pacing Model Establishment in Rabbits with AF

In this study, the pacing mode was AOO (atrium is paced at a set rate regardless of atrial activity) with 600 beats/min. The rabbits had a normal rhythm and pacing rhythm. The normal rhythm was regular, and the frequency was approximately 250 ± 15 beats/min (Figure 1(a)). The pacing rhythm was irregular and fast, approximately 600 ± 23 beats/min (Figure 1(b)).

Sac/val treatment effect upon AERP in rabbits was studied. The AERP_150_ ms values of rabbits in the control cohort, pacing cohort, and sac/val + pacing cohort were identified. AERP_150_ for the control cohort was 116 ms (Figure 2(a)). The AERP_150_ for the pacing cohort was 64 ms (Figure 2(b)). The AERP_150_ for pacing+sac/val cohort was 99 ms (Figure 2(c)). The AERP_150_ values of the control cohort, pacing cohort, and pacing+sac/val cohort were statistically analyzed and compared. In comparison with the control cohort, AERP_150_ was markedly decreased within the pacing cohort (*P* < 0.05). In comparison with the pacing cohort, AERP_150_ was markedly increased within the pacing+sac/val cohort (*P* < 0.05). AERP_150_ was markedly reduced in the pacing cohort followed by the control cohort. Sac/val treatment rescued such reductions in AERP_150_ (Figure 2(d)).

Sac/val therapeutic function upon inducibility rate for AF was studied. AF occurrences in rabbits of the control cohort, pacing cohort, and pacing+sac/val cohort were detected. According to our results, AF was not induced within the control cohort (Figure 3(a)) and induced within the pacing cohort (Figure 3(b)). Inducibility rates of AF within the control cohort, pacing cohort, and pacing+sac/val cohort were statistically analyzed and compared. In comparison to the control cohort, the AF inducibility rate was markedly increased in the pacing cohort (*P* < 0.05). In comparison to the pacing cohort, the AF inducibility rate was markedly decreased in the pacing+sac/val cohort (*P* < 0.05). The rabbits in the pacing cohort showed a stronger indication of AF than animals in the control cohort. However, in comparison with the pacing cohort, AF incidence was lowered within the sac/val-treated cohort (Figure 3(c)).

### 3.2. Regulation for CaMKII/Ca_v_1.2 Signaling Pathway *In Vivo* and in a Rapid Electrical Stimulation Model *In Vitro*

Sac/val regulated the CaMKII-Ca_v_1.2 signaling pathway in rabbits' AF model. The CaMKII and Ca_v_1.2 protein levels in the control cohort, pacing cohort, and pacing+sac/val cohort were analyzed and compared. Our results showed that the Ca_v_1.2 protein level was markedly reduced whereas that of the CaMKII was strongly increased in the pacing cohort when compared with the control cohort (*P* < 0.05). The proteomic levels of Ca_v_1.2 were markedly upregulated whereas the levels of CaMKII were downregulated in the pacing+sac/val cohort when compared with the pacing cohort (*P* < 0.05), and sac/val reversed the changes of both proteins (Figures 4(a)–4(d)). Similarly, in the high-frequency electrical stimulation (pacing) model of HL-1 cultures, the Ca_v_1.2 expression was severely downregulated, whereas CaMKII levels were markedly upregulated in the pacing cohort in comparison with the control cohort (*P* < 0.05). The proteomic expression of Ca_v_1.2 was markedly upregulated, while CaMKII was severely downregulated in the pacing+sac/val cohort in comparison with the pacing cohort (*P* < 0.05), and the changes were inhibited through LBQ657 and valsartan (Figures 4(e)–4(h)). Sac/val regulated the CaMKII/Ca_v_1.2 expression in HL-1 culture and rabbit models of rapid electrical stimulation.

## 4. Discussion

This investigation demonstrated that sac/val regulated the CaMKII/Ca_v_1.2 signaling pathway in atrial rapid electrical stimulation models. Previous studies have shown that rapid atrial pacing can activate CaMKII, which modulates L-type calcium channel opening by enhanced phosphorylation of the Ca_v_1.2 channel and promotes AF atrial electrical remodeling [9], typically exhibiting atrial electrical remodeling through AERP reduction, as well as downregulation of Ca_v_1.2 protein expression, whereby lowering *I*CaL shortens the APD and finally promotes the occurrence of AF [8, 31, 32]. Previous studies have confirmed that the natriuretic peptide (NP) family can improve electrical remodeling in AF [11]. Sac/val attenuated AF electrical remodeling through lowering AF inducibility and circumventing diminished AERP, probably via the CaMKII/Ca_v_1.2 pathway. Such dataset outcomes corroborate with past results, discovering that sac/val alleviated these changes in AF models via the CaMKII/Ca_v_1.2 pathway.

### 4.1. CaMKII/Ca_v_1.2 Signaling Pathway in AF

A study of dementia showed that CaMKII and Ca_v_1.2 protein expression within CaMKII/Ca_v_1.2 signaling pathway exhibits an opposite trend in a mouse model [33]. However, there is no evidence that the CaMKII/Ca_v_1.2 signaling pathway exists within the myocardium. A previous study showed proteomic levels for CaMKII and Ca_v_1.2 in the AF model with opposing trends [32] which was consistent with the trend of CaMKII and Ca_v_1.2 protein expression within the above research on dementia. Therefore, we speculate that the CaMKII/Ca_v_1.2 signaling pathway exists within the atrial myocardium.

### 4.2. Role of the CaMKII/Ca_v_1.2 Pathway in Electrical Remodeling of AF

Ca_v_1.2 is a subtype of LTCCs within the myocardium that has a pivotal role in action potential formation, triggering excitation/contraction in cardiomyocytes [34]. CaMKII is a serine/threonine kinase having a key role in multiple cardiac remodeling functions, such as ion-channel gene expression modulation [35, 36]. CaMKII, as an upstream protein regulating LTCCs, can phosphorylate Ca_v_1.2 and decrease its expression [9]. These changes lead to electrical reconfiguration, including the shortening of AERP, ultimately promoting the occurrence and maintenance of AF [37]. Therefore, we evaluated the AERP and CaMKII and Ca_v_1.2 protein levels. We found that the AF induction rate was markedly increased, the AERP was markedly reduced after 3 weeks' rapid pacing, CaMKII expression was increased, and Ca_v_1.2 expression was decreased. CaMKII expression was markedly upregulated while Ca_v_1.2 was markedly downregulated within HL-1 cultures.

### 4.3. Sac/Val Regulated the CaMKII/Ca_v_1.2 Pathway in AF Electrical Stimulation Models

Sac/val can inhibit the degradation of NPs and thus increase their levels. Past investigations revealed that NPs attenuate atrial electrical remodeling in AF. Atrial myocytes express ANP genes [38], and mutant atrial NP (Mut-ANP) promotes ion channel remodeling in familial AF [39]. An investigation indicated Ang-(1–7) to prevent cardiac electrical remodeling induced by ARP in dogs by increasing ANP secretion [40]. Atrial myocytes also express B-type natriuretic peptide (BNP) genes, with atria being predominating sources for BNP in “lone AF” [41]. Long-term BNP therapeutics prevented atrial electrical remodeling in AF-rabbit models [11]. BNP and CNP can increase the *I*CaL of right atrial myocytes by activating NP receptors, thus increasing the spontaneous action potential frequency of isolated mouse cardiomyocytes [42]. The CNP level was markedly upregulated in AF cases [43]. The above results indicate that sac/val can reduce atrial electrical remodeling in AF cases by increasing the levels of NPs.

A previous study showed that treatment with valsartan can alleviate atrial electrical remodeling in AF [44]. Sac/val had increased effectiveness for ameliorating left atrial (LA)/LA appendage (LAA) activity, in comparison to ARBs (angiotensin receptor blockers) within humans/murines [45]. Other studies have shown that sac/val has a stronger effect than ACEIs or ARBs in myocardial infarction and HF [17, 18, 46, 47]. Our study found that sac/val regulated the CaMKII/Ca_v_1.2 pathway in atrial rapid electrical stimulation models, but additional research is required to validate increased effectiveness in comparison with valsartan.

Studies have shown that BNP can effectively improve atrial electrical remodeling in animal models of AF through the CaMKII pathway and reduce the incidence of AF [11]. Recent research demonstrated that sac/val can inhibit atrial remodeling in AF through the CaN/NFAT pathway [48]. Such an endpoint corroborated with this investigation's dataset outcomes. We found that sac/val effectively regulated the CaMKII/Ca_v_1.2 expression and could alter this pathway in atrial rapid electrical stimulation models. Therefore, the above-described investigation could contribute to a novel strategy in AF therapeutics in clinical settings.

## 5. Study Limitations

First, our observations are derived from a rabbit model for AF driven through fast atrial pacing. However, clinical AF is often complicated by valvular/coronary heart disease/HF/hypertension, and solitary AF can also occur. This rabbit model simulates “lone AF” and does not fully reflect complex clinical spectra within human AF. Secondly, NPs have many physiological functions and can protect the heart through various mechanisms. Such an investigation was restricted to observing sac/val influence upon calcium regulation for the CaMKII/Ca_v_1.2 signaling pathway within the AF model and did not examine sac/val influence upon atrial electrical remodeling, structural and autonomic nerve remodeling, or AF-related intracellular calcium-handling remodeling. The lack of histological analyses is another limitation. Third, this study did not establish a rapid pacing + valsartan cohort and never compared sac/val and valsartan influence in AF. Fourth, the species used within *in vivo* assays varied from *in vitro* assays.

## 6. Conclusion

The sac/val is gaining wider research interests these days for various cardiac-related pathway regulation. This study was designed to validate sac/val influence on CaMKII/Ca_v_1.2 expression in rabbit model and HL-1 AF cultures. The AF induction rate was markedly increased together with AERP reduction in the pacing cohort. The sac/val treatment rescued such changes in pacing+sac/val cohort. The proteomic expression profiles of CaMKII and Ca_v_1.2 showed that the CaMKII expression was markedly upregulated, while Ca_v_1.2 expression was downregulated in the pacing cohort. These effects were absent in the pacing+sac/val cohort. Results of this study showed that sac/val can affect the CaMKII/Ca_v_1.2 expression and thus could lead to altering the CaMKII/Ca_v_1.2 signaling pathway in the atrial fibrillation stimulation rabbit model. In the future, further research is needed to establish and validate the role of sac/val on the CaMKII/Ca_v_1.2 pathway regulation to prevent and treat atrial fibrillation with sac/val.

## Figures and Tables

**Figure 1:** Comparison of the pacing of rabbits through electrocardiogram (ECG): (a) rabbits within the normal cohort and (b) rabbits within the pacing cohort.

**Figure 2:** Representation of AERP_150_ ms values for rabbits in (a) the control cohort (116 ms), (b) the pacing cohort (64 ms), (c) the pacing+sac/val cohort (99 ms), and (d) shows statistical analysis results for AERP_150_ values of control cohort, pacing cohort, and pacing+sac/val cohort. ^∗^*P* < 0.05 for comparison of pacing cohort with a control cohort. ^#^*P* < 0.05 for comparison of pacing+sac/val cohort with pacing cohort.

**Figure 3:** Representation of the typical ECG of animal (a) without AF induction, (b) ECG of animal with induced AF, and (c) comparison of AF inducibility between control cohort, pacing cohort, and pacing+sac/val cohort. ^∗^*P* < 0.05 represents the comparison of the pacing cohort with the control cohort. ^#^*P* < 0.05 represents the comparison of the pacing+sac/val cohort with the pacing cohort.

**Figure 4:** Representation of the changes in Ca_v_1.2 and CaMKII levels in rabbits and HL-1 cultures where (a) and (b) show the Ca_v_1.2 protein levels in rabbits of three cohorts. ^∗^*P* < 0.05 represents the comparison of the pacing cohort with the control cohort. ^#^*P* < 0.05 represents the comparison of the pacing+sac/val cohort with the pacing cohort. (c, d) The CaMKII protein levels in rabbits from the three cohorts. ^∗^*P* < 0.05 for comparison of pacing cohort with a control cohort. ^#^*P* < 0.05 for comparison of the pacing+sac/val cohort with the pacing cohort. (e, f) The Ca_v_1.2 protein levels in HL-1 cultures for three cohorts. ^∗^*P* < 0.05 for comparison of pacing cohort with control cohort and ^#^*P* < 0.05 for comparison of pacing+sac/val cohort with pacing cohort. (g, h) The CaMKII protein levels in HL-1 cultures for three cohorts. ^∗^*P* < 0.05 for comparison of pacing cohort with a control cohort. ^#^*P* < 0.05 for comparison of the pacing+sac/val cohort with the pacing cohort.

## Data Availability

Data will be provided on request.
